# Complications associated with transobturator sling procedures: analysis of 233 consecutive cases with a 27 months follow-up

**DOI:** 10.1186/1472-6874-9-28

**Published:** 2009-09-25

**Authors:** Isabelle Kaelin-Gambirasio, Sandrine Jacob, Michel Boulvain, Jean-Bernard Dubuisson, Patrick Dällenbach

**Affiliations:** 1 Department of Gynecology and Obstetrics, Division of Gynecology, Perineology Unit, University Hospitals of Geneva, University of Geneva, Switzerland; 2 Department of Gynecology and Obstetrics, Division of Obstetrics, Clinical Research Unit University Hospitals of Geneva, University of Geneva, Switzerland

## Abstract

**Backround:**

The transobturator tape procedure (TOT) is an effective surgical treatment of female stress urinary incontinence. However data concerning safety are rare, follow-up is often less than two years, and complications are probably underreported. The aim of this study was to describe early and late complications associated with TOT procedures and identify risk factors for erosions.

**Methods:**

It was a 27 months follow-up of a cohort of 233 women who underwent TOT with three different types of slings (Aris^®^, Obtape^®^, TVT-O^®^). Follow-up information was available for 225 (96.6%) women.

**Results:**

There were few per operative complications. Forty-eight women (21.3%) reported late complications including *de novo *or worsening of preexisting urgencies (10.2%), perineal pain (2.2%), *de novo *dyspareunia (9%), and vaginal erosion (7.6%). The risk of erosion significantly differed between the three types of slings and was 4%, 17% and 0% for Aris^®^, Obtape^® ^and TVT-O^® ^respectively (P = 0.001). The overall proportion of women satisfied by the procedure was 72.1%. The percentage of women satisfied was significantly lower in women who experienced erosion (29.4%) compared to women who did not (78.4%) (RR 0.14, 95% CI 0.05-0.38, P < 0.001).

**Conclusion:**

Late post operative complications are relatively frequent after TOT and can impair patient's satisfaction. Women should be informed of these potential complications preoperatively and require careful follow-up after the procedure. Choice of the safest sling material is crucial as it is a risk factor for erosion.

## Background

Urinary incontinence is a major public health problem. In Europe, it is estimated to affect up to one third of women older than the age of 18 years. The prevalence increases with age and reaches 45% at 60 years [1]. In 1995, the tension-free-vaginal-tape (TVT) procedure was introduced and has revolutionized the surgical treatment of female stress urinary incontinence (SUI) due to its simplicity, efficiency and minimal invasiveness [2]. However patients can be exposed to several complications [3]. One category of complications is associated with the blind passage of the tape through the retropubic space causing bladder or bowel perforation, or vascular injuries. The other category is related to voiding disorders such as dysuria, or *de novo *urgency. In a quest to find a minimally invasive sling associated with even less morbidity than the TVT, the transobturator tape (TOT) was created [4] and a modified procedure (TVT-O) was reported by de Leval [5]. Since its introduction numerous reports confirmed its effectiveness with an objective and a subjective cure rate up to 80% and 92% respectively and low morbidity [6,7]. However, complications are probably underreported [8]. Recently few articles reported high erosion rates [9,10], ischio rectal abcess [11,12] as well as other complications. Data concerning safety are rare, follow-up is often less than two years, and risk factors for erosions are poorly described [13].

The aim of this study was to describe the complications, and especially late ones, associated with the transobturator sling procedure. One specific objective was to identify risk factors for erosions.

## Methods

We included 233 consecutive women who had undergone transobturator sling procedure for pure stress or mixed urinary incontinence in the Department of Obstetrics and Gynecology, Geneva University Hospitals, from June 2003 to October 2006. This study was approved by the Institutional Ethics Committee of the Geneva University Hospitals. We collected Variables including age, weight, height, menopausal status, hormonal replacement therapy, previous hysterectomy or genital prolapse surgery. Urodynamics was systematically performed preoperatively, according to the standards recommended by the International Continence Society[14]. In women with concomitant urge incontinence, causes were searched and treated. All women had a standardized preoperative prolapse assessment using Baden-Walker classification[15]. The operative technique used was based on Delorme's description [4] for the outside-in technique and on De Leval's [5] for the inside-out technique. Cystoscopy was not systematically performed. We used three different types of slings during the study period: ObTape^® ^(Mentor-Porges, Le Plessis Robinson, France), TVT-O^® ^(Gynecare, Johnson and Johnson, Spreitenbach, Suisse) and Aris^® ^(Porges, Le Plessis Robinson, France). Surgery was performed by six senior surgeons. Prophylactic antibiotics (cefoxitin 2 g intravenously) was systematically administered.

Data about surgery, the type of sling procedure, associated surgery, per-operative and early postoperative complications were collected in the charts. The follow up period after TOT ranged from 5 to 50 months. Follow-up included for all patients a clinical examination one month after surgery by their surgeon. We also recorded data on any assessment made during the study period in our department. Per operative complications (vaginal perforation, haemorrhage, vesical or urethral perforation), early post-operative complications (hematoma, dysuria, infection) and late post-operative complications (erosions, ischio-rectal abscess, perineal pain, *de novo *dyspareunia, *de novo *urge or impaired urge incontinence) were searched. In case of urgencies, infection was excluded by urine analysis. Early post-operative period was defined as from one day to one month after surgery and late post-operative period more than one month.

In addition, between the first of September 2007 and the 31st of December 2007 all women were contacted by telephone by one of the investigators (IKG) and asked standardized questions to complete the assessement of late post-operative complications.

Means were compared with the t-test and proportions with the chi-square test. A P value less than or equal to 0.05 was considered to be statistically significant and 95% confidence intervals (CIs) were reported. We performed a univariable analysis to compute the relative risks and their 95% CI, for each predictor of erosions. Mean intervals from TOT procedure to events (erosion or end of follow-up) were estimated for each type of sling from life tables (Kaplan-Meier), and survival curves were compared by the Peto log-rank test. The Cox model was used to calculate hazard ratios (HRs) to adjust for the different duration of follow-up with the various slings. Data were managed and analyzed with SPSS 15.0 statistical software (SPSS Inc., Chicago, IL).

## Results

Between June 2003 and December 2006, we performed 233 transobturator sling procedures for the treatment of female stress incontinence in our institution. The characteristics of the patients are reported in Table 1. The mean follow-up was 27 months (SD = 9.7). Fifty-eight (24.9%) patients had the TOT under loco-regional and 175 (75.1%) under general anaesthesia. TOT was the only procedure in 129 patients and was associated with another surgical intervention in 104 women (11 total laparoscopic hysterectomies, 33 vaginal hysterectomies, 58 vaginal anterior repairs, 53 vaginal posterior repairs, 21 vaginal vault suspensions to the sacrospinous ligament according to Richter, and 22 other procedures such as conisation, laparoscopy and hysteroscopy). The indication for TOT was stress incontinence with pure stress incontinence in 153 (65.7%) and mixed urinary incontinence in 80 women (34.3%). The mean hospitalization duration was 3.5 days (range 1 to 19 days). For women who had only TOT procedure, the mean hospitalization stay was 2.2 days (range 1 to 6 days) compared to 5.2 days (range 2 to 19 days) for women who had other surgical procedure associated with the TOT (P < 0.001).

**Table 1:** Characteristics of the study population

**Characteristics**	**Total N = 233**
Age (y) mean (SD)	57.9 (13.2)
Height (cm) mean (SD)	1.60 (0.06)
Weight (kg) mean (SD)	70.7 (14)
BMI (kg/m^2^) mean (SD)	27.6 (5)
Menopause n (%)	156 (67)
HT n (%)	52 (22.3)
	
Menopause without HT n (%)	104 (44.6)
Pure stress incontinence n (%)	153 (65.7)
Mixed urinary incontinence n (%)	80 (34.3)
Previous hysterectomy n (%)	40 (17.2)
Previous prolapse surgery n (%)	31 (13.3)
Sexual Activity n (%)	156 (67)

BMI = body mass index; HT = hormonal replacement therapy

We used three types of slings: Aris^® ^in 101 (43.4%), Obtape^® ^in 76 (32.4%) and TVT-O^® ^in 56 (24.0%) women. The mean follow-up was 18.8 months (SD = 4.5), 34.3 months (SD = 8.4), and 33.3 months (SD = 5.7) for Aris^®^, Obtape^® ^and TVT-O^® ^respectively (P < 0.001).

Six women were lost to follow-up (2 TVT-O^®^, 2 Obtape^® ^and 2 Aris^®^) and two had died (1 TVT-O^®^, 1 Obtape^®^) at phone contact, leaving 225 women available for the late post-operative analysis. The complications are reported in table 2 and divided in per-operative complications, early postoperative and late postoperative complications. Peroperative complications were very rare apart from bleeding more than 200 ml which occurred in 12 women (5.2%), 8 times in women with TOT only and 4 times in women with another additional surgical procedure. However none of the patients required blood transfusion. There was no bladder perforation. Seven women (3%) had urinary retention after surgery. Retention lasted less than 72 hours for five of them (2.1%) and was successfully treated using a Foley catheter. Retention lasted more than 72 hours for two women (0.9%). One of them needed section of the sling and the other one needed intermittent self catheterization during 15 days.

**Table 2:** Complications

**Complications**	**Total** **N = 233**	**Obtape^®^** **N = 76**	**Aris^®^** **n = 101**	**TVT-O^®^** **n = 56**	**P value**
During procedure n (%)					
Haemorrhage>200 ml	12 (5.2)	2 (2.6)	9 (8.9)	1 (1.8)	0.07
Vaginal perforation	2(0.9)	0	2 (2.0)	0	0.27
Bladder perforation	0 (0)	0	0	0	NA
					
Early-postoperative n (%)					
Urinary retention	6 (2.6%)	3 (3.9)	1 (1.0)	2 (3.6)	0.41
Section of the sling	1(0.4%)	0	0	1 (1.8)	0.21
Haematoma	1(0.4%)	0	0	1 (1.8)	0.21
					
Late post-operative* n (%)					
Vaginal erosions	17 (7.6%)	13 (17.8)	4 (4.0)	0	>0.001
Reintervention^†^	14 (6.2%)	11 (15.1)	3 (3.0)	0	0.001
Abscess	1 (0.4%)	1 (1.4)	0	0	0.35
*De novo *dyspareunia	14 (6.2%)	7 (9.6)	5 (5.1)	2 (3.8)	0.33
*De novo *urgency	14 (6.2%)	8 (11.0)	2 (2.0)	4 (7.5)	0.05
Perineal pain	5 (2.2%)	2 (2.7)	2 (2.0)	1 (1.9)	0.93
Worsening of urgency	9 (4.0%)	3 (4.1)	3 (3.0)	3 (5.7)	0.73

P values are calculated with the chi-squared test

*Percentage are calculated with N = 225 (73 Obtape^®^, 99 Aris^®^, 53 TVT-O^®^)

^†^Reinterventionfor vaginal erosion

There was no difference in term of per operative and early post operative complications between women who had TOT procedure in addition with another surgical procedure compared to women who had TOT only (RR 0.93, 95% CI 0.64-1.34, P = 0.71).

Overall late complication rate was 21.3% (48/225 women). There was no difference between women who had concomitant procedures and women who had TOT as an only surgical procedure (RR 0.86, 95% CI 0.59-1.27, P = 0.45). Late postoperative complications were *de novo *urgency in 14 patients (6.2%), perineal pain in five (2.2%) and aggravation of urge incontinence in nine (4%). Dyspareunia *de novo *occurred in 14 patients of the 156 sexually active women (9%). As above, there was no difference between women who had combined procedures and women who had solitary TOT's for specific late complications. Seventeen patients developed vaginal erosions (7.6%) among which one developed an abscess of the obturator fossa 38 months after insertion of the sling. Drainage of the gluteal abscess was performed followed by removal of the vaginal mesh and antibiotics were administered intravenously for five days and completed for ten days orally. The patient was discharged after one week. At follow-up five months later, the woman was asymptomatic and without incontinence. The mean time from TOT procedure to diagnosis of erosion was 11 months (range 1 to 37 months). Fourteen of the 17 women with erosion (82.4%) required reintervention with section and total or partial removal of the sling. Three of them (17.6%) were successfully treated conservatively with local estrogens and antiseptic treatment. The size of erosion was less than one centimeter and healing was achieved in four to 10 weeks. The proportion of erosions was significantly different between the three types of slings. There were four erosions in women treated with Aris^® ^(4%) compared to 13 erosions in the Obtape^® ^group (17.8%) (RR 0.23, 95% CI 0.08-0.67, P = 0.003). There was no erosion in the TVT-O^® ^group (Table 2). The difference between TVT-O^® ^and Aris^® ^groups was not statistically significant (P = 0.17). The mean interval from TOT procedure to diagnosis of erosion was 8.8 months (range 2 to 17 months) for Aris^® ^and 11.7 mo (range 1 to 37 months) for Obtape^® ^(P = 0.6) respectively. The mean age and BMI were similar in women with erosion compared to women who did not present with erosion during the study period. In time to event analysis, the difference between the three slings was statistically significant (log-rank test 0.001) (Fig. 1). After adjustment for the duration of follow up in a Cox model, the hazard ratio still showed a decreased risk of erosion in the Aris^® ^compared with the Obtape^® ^group (HR 0.27, 95% CI 0.09-0.86; p = 0.03). Apart from the type of sling, we did not identify any other significant risk factor of erosions (Table 3).

**Table 3:** Comparisons between women with and without erosions (N = 225)

**Predictor**	**Erosions** **(n = 17)**	**No erosions** **(n = 208)**	**Relative risk** **(95% CI)**	**P value**
Type of sling n (%)				
Obtape^®^	13 (76.5)	60 (28.8)	Réf.	
Aris^®^	4 (23.5)	95 (45.7)	0.23 (0.08-0.67)	0.003
TVT-O^®^	0	53 (25.5)	NA	0.001
Haemorrhage > 200 ml n (%)	2 (5.9)	10 (4.8)	2.37 (0.61-9.18)	0.22
Sexual activity n (%)				
No	4 (23.5%)	65 (31.3%)	Réf.	
Yes	13 (76.5%)	143 (68.8%)	1.44 (0.49-4.25)	0.51
Age: mean (SD)	58.0 (13.4)	56.9 (12.3)	NA	0.35
BMI: mean (SD)	27.6 (1.2)	27.7 (0.4)	NA	0.39
Concomitant surgery n (%)				
None	9 (52.9)	116 (55.8)	Réf.	
Prolapse surgery	3 (17.6%)	72 (34.6%)	0.56 (0.16-1.99)	0.36
Hysterectomy	1(5.9)	41 (19.7%)	0.33 (0.04-2.53)	0.26
Any surgery	8 (47.1)	92 (44.2)	1.11 (0.44-2.78)	0.82
Hypoestrogeny n (%)				
No	12 (70.6%)	111 (53.4%)	Réf.	
Yes	5 (29.4%)	97 (46.6%)	0.88 (0.26-2.95)	0.84

P values are calculated with the chi-squared test for proportions and with the T-test for means unless specified.

**Figure 1:** **Survival analysis comparing Aris^®^, Obtape^® ^ant TVT-O^® ^slings for the occurrence of vaginal erosion**.

The overall proportion of women satisfied by the procedure was 72.1%. The percentage of women satisfied was significantly lower in women who experienced erosion (29.4%) compared to women who did not (78.4%) (RR 0.14, 95% CI 0.05-0.38, P < 0.001). Satisfaction was significantly reduced in women who developed *de novo *dyspareunia (42.9%) and *de novo *urgency (35.7%) compared to those who did not (76.8% and 77.3%, respectively) (RR 0.25, 95% CI 0.09-0.70, P = 0.005 and RR 0.19, 95% CI 0.07-0.54, P < 0.001, respectively). Satisfaction was also reduced in the five women reporting perineal pain (40%) compared to those who did not (75.5%) (RR 0.53, 95% CI 0.18-1.56, P = 0.07).

## Discussion

Our study confirms that at short term, TOT is a safe procedure with very few per-operative and early post operative complications. However, during the long term follow-up, occurrence of *de novo *urge symptoms, *de novo *dyspareunia, perineal pain, and vaginal erosions significantly reduced the satisfaction of patients.

The only relevant per-operative complication, in our study, was haemorrhage of more than 200 ml (5.2%), but there were no haematomas, and no transfusion was required. Different series of TOT procedures report similar risks of bleeding rates varying between 0.83 and 5.4% [16,17]. In a large study the incidence of intra operative bleeding of more than 200 ml was 1.9% for the TVT procedure [3].

The incidence of urinary retention is low in our study and is similar to the rates of 1.5% reported by other authors [7,16]. In a recent review [18] which compared retropubic and transobturator tapes, voiding lower urinary tract symptoms were less common with the transobturator route.

*De novo urge *symptoms have a high impact on quality of life [19]. We observed 6.2% of women with persistent *de novo *urgency at long term follow-up which is similar to other studies [17,20]. In comparison, the risk with TVT is reported to be higher in the short term (33% for TVT vs 8% for TOT) [21], but after a longer follow up period, the risk is similar (6.3%) [22].

In our study, most women were sexually active (67%) and among them 9% reported *de novo *dyspareunia after the operation. This complication has a potential high impact on the quality of life, as the overall proportion of women satisfied with the procedure drops dramatically when it occurs (76.8% compared to 42.9%, P = 0.005). In a recent study [17], dyspareunia was more frequent after TOT (19.2% compared to 16.2% before), but the finding was not considered statistically significant. In another study, dyspareunia was reported in eight over 78 sexually active women (10.3%) [6]. After TVT no significant difference in the incidence of dyspareunia was found post-operatively [23].

Perineal pain is reported to occur in 2.3% to 5% after transobturator surgery, to be transient, resolving within the first month [16,24]. We report the same rates, but with persistent pain on long term follow up. The risk of groin pain is higher with TOT and TVT-O, compared to the TVT (OR 8.28, 95% CI 2.7-25.4) [25].

In our study 17 women had vaginal erosions. The proportion of women satisfied with the procedure was significantly reduced when erosion occurred. The mean time to erosions varied, which emphasizes the need to pay attention when symptoms like vaginal discharge, pain or dyspareunia occur even after a long period. Since some erosion occur without symptoms and can not be detected through telephone contact, this complication might be underestimated in our study. The majority of women who developed erosions required a reintervention. One woman presented with an abscess of the obturator fossa 38 months after surgery. In a recent review of suburethral sling procedures complications [26], the frequency of erosions after TOT varied between 1.8% and 20.0%. In a recent meta-analysis [25], erosions were more common after tape insertion by the transobturator route (TVT-O and TOT) compared to the retropubic route (OR 1.96; 95% CI 0.87-4.39). After a systematic search in the Manufacturer and User Facility Device Experience Database (MAUDE), Boyles et al. concluded that erosions constituted 60% of the complications associated with the TOT and are probably underreported [27]. In our analysis the only significant risk factor for erosion was the type of sling, with a very high risk (17.8%) for the Obtape^® ^sling compared to the two others. The mean follow-up was different between the three types of slings. However, the difference in the occurrence of erosion remained significant after adjustment for the duration in a multivariable model. There were more per operative complications with Aris^® ^(12) than with Obtape^® ^(5) which suggest that per operative complications were not a risk factor for the development of vaginal erosions.

We believe that vaginal erosion might be secondary to three potential factors: the sling material, surgical technique, or individual patient factors. Our data confirm that the tolerance of vaginal tissue depends on the type of sling used. The three tapes used in our study are polypropylene monofilaments. The TVT-O^® ^and Aris^® ^slings are type I meshes because they are macroporous (>75 *μ*m). The Obtape^® ^sling is more of a type II mesh since the pores are smaller (50 *μ*m). The incidence of erosion with this sling was very high in our study which is similar to that of other studies if duration of follow up is taken into account [9,10,28]. As the Obtape^® ^sling carries an important risk of vaginal erosion, we have abandoned its use. Type I mesh is considered to limit the risk of erosions [13,29] because of a lower risk of infection, a lower inflammatory response and a better incorporation in the surrounding tissue. Aris^® ^and TVT-O^® ^are both type I meshes, but they have different mechanicals characteristics (different sizes of pores, different elasticity). No erosions were diagnosed after TVT-O^®^, but the number of women was small. Other authors also reported a low risk using this device (0.9%-1.8%) [10,30].

Another difference between Aris^® ^and TVT-O^® ^is the surgical technique, TVT-O^® ^being an in-out procedure and Aris^® ^an out-in one. However, there was no statistically significant difference for the risk of erosion between the two techniques in our study and we are not able to determine if the surgical technique itself plays a role in the risk of erosion. We found only one study in which the authors concluded that erosion rate was associated with the surgical technique. They showed that plicaturing the pubocervical fascia between the sling and the vaginal mucosa could reduce the occurrence of erosion [31].

Individual patient characteristics (age, estrogen status, concomitant surgery, sexual activity) may play a role in the occurrence of vaginal erosion. Unfortunately, our study does not have the power to show differences in these potential risk factors. A study reported that diabetes mellitus was the only individual patient characteristic to be associated with a higher risk of erosions (RR 8.3, 95% CI 1.6-43.0) [13].

The strength of this study was the availability of a continuous cohort of women with a mean follow-up of more than two years and few patients lost for follow-up (6/233, 2.6%).

The limitations of our study included those typical of studies relying on information collected using medical files and during a telephone contact, with the risk of information bias. To avoid these biases, standardized questions were asked to the patients. Our evaluation of satisfaction was limited by the fact that we asked women their views by telephone without using a more detailed questionnaire. TOT was accompanied by another surgical procedure in almost half of the cases which could confound the analysis. However, this is not the case, because there was no difference in the occurrence of early or late complications between women with or without concomitant other surgical procedure.

## Conclusion

Late post operative complications are relatively frequent after TOT and can impair patient's satisfaction. Women should be informed of these potential complications preoperatively and require careful follow-up after the procedure. Choice of the safest sling material is crucial as it is a risk factor for erosion.

## Abbreviations

BMI: body mass index; HT: hormonal replacement therapy; TOT: transobturator tape; TVT: retropubic transvaginal tape; TVT-O: inside-out transobturator tape; SUI: stress urinary incontinence

## Competing interests

The authors declare that they have no competing interests.

## Authors' contributions

IKG was involved in study design, data collection, data analysis and manuscript writing. SJ participated in the conception and design of the study, and in revising the manuscript. MB participated in the analysis and interpretation of data and in revising the manuscript. JBD was involved in the conception and design of the study and in revising the manuscript. PD was involved in study design, analysis and interpretation of data, and manuscript writing. All authors read and approved the final manuscript.

## Pre-publication history

The pre-publication history for this paper can be accessed here:


